# The Function Mechanism of the Current Situation of Chinese Cultural Integration and Environment on the Development of Chinese Enterprises

**DOI:** 10.1155/2022/4393337

**Published:** 2022-06-17

**Authors:** Shuwen Zhang

**Affiliations:** Law School and Intellectual Property School, Jinan University, Guangzhou 510632, China

## Abstract

China's economy is booming and many Chinese enterprises are growing rapidly. The report card handed over by Chinese enterprises through practical actions proves that Chinese outstanding entrepreneurs have successful modern management experience. These Chinese entrepreneurs have experienced the test of practice, and the experience gained has Chinese characteristics and is worth promoting. Entrepreneurs carry out more business management practices, which also provides valuable reference resources for the study of Chinese management thought. At the same time, *The Times* is also calling for more Chinese entrepreneurs to form their own management ideas. The influence of the current situation of the Chinese cultural integration environment on the development of Chinese enterprises is mainly that a good cultural integration environment will promote the development of enterprises and provide preconditions for the development of Chinese enterprises. This paper studies the current situation of Chinese culture integration environment of Chinese entrepreneur management thought formation process; the main purpose is, through the analysis of Chinese outstanding entrepreneur management thought formation process, to reveal the Chinese culture integration management environment formation law and essential characteristics, in order to enrich the management cognitive research and Chinese entrepreneurs management thought research, publicity, and promotion of Chinese outstanding entrepreneurs form management thought and also to provide a reference for more practitioners.

## 1. Introduction

The Chinese nation is a nation with strong cohesion and centripetal force. This cohesion and centripetal force largely stems from the Chinese nation's high recognition of Chinese culture. In recent years, the economic strength of overseas Chinese has continued to grow, and Chinese enterprises have changed from labor-intensive to capital- and technology-intensive. The contribution of overseas Chinese to China's economic development has also been continuously affirmed and emphasized. The thesis aims to explore the development of overseas Chinese culture in Chinese enterprises. First of all, we need to interpret these two terms: Chinese refers to former Chinese citizens and their descendants of foreign nationality [1], who have joined the nationality of other countries; overseas Chinese refers to Chinese citizens residing abroad who have Chinese nationality [1]. Overseas Chinese culture is a complex combination of traditional agricultural civilization and rationalist cultural spirit dominated by modern industrial civilization [2]. It includes both traditional agricultural civilization and rationalist cultural spirit dominated by modern industrial civilization. After World War II, the society of overseas Chinese has changed, which is also the most far-reaching change in the history of overseas Chinese. More than 90% of overseas Chinese have joined local nationality and slowly integrated into the local environment politically, economically, and culturally. At the same time, it also brought Chinese culture to the local area. Chinese culture began to change slowly, and overseas Chinese culture gradually formed. The gradual commercialization of overseas Chinese culture, coupled with the local socioeconomic and political recognition from overseas Chinese to overseas Chinese, has undoubtedly accelerated the localization process of overseas Chinese [3]. The so-called overseas Chinese culture is essentially a Chinese culture transplanted overseas and preserved among overseas Chinese, which belongs to “overseas Chinese culture.” In today's social, economic, and cultural context, it can be found that overseas Chinese going abroad is different from the colonialism of Western countries under the protection of power, but peaceful and civilized immigration with working people as the main body. The overseas Chinese culture is relatively independent, highlighting the spirit of Chinese enterprises.. At the same time, it is also the product of the combination of Chinese and Western cultures. It has not been assimilated into the development process of the world but can develop and innovate in the torrent of economic exchanges and cultural torrents, maintain a free development method, and become a driving force. The driving force for the further development and self-improvement of the overseas Chinese culture, thus spawning a group of overseas Chinese with a higher level of knowledge and strong adaptability, making contributions in the fields of economy, culture, science, and technology. Development opportunities for Chinese Enterprises: “the Belt and Road” International Cooperation Summit Forum. The opening of the forum at the Beijing National Convention Center has attracted the attention of overseas Chinese all over the world and also made overseas Chinese in other countries feel the opportunities and honors of the motherland. After the efforts and accumulation of several generations of overseas Chinese, batches of overseas Chinese businessmen with strong capital strength and economic resources have seen new opportunities for career development and life under the “Belt and Road” initiative by virtue of their unique advantages of “connecting China and foreign countries.” The interactive relationship between Chinese enterprises and overseas Chinese is conducive to the implementation of the “Belt and Road” initiative and jointly promotes the economic cooperation between my country and the countries along the “Belt and Road.” Simultaneously, from the existing research results, there are many definitions of the corporate culture. Although there are differences in views and expressions, there is also a basic consensus that the core of corporate culture is set as values or related expressions (see Table 1).

## 2. Cultural Characteristics of Overseas Chinese

As shown in Figure 1, in today's socioeconomic and cultural context, it can be found that overseas Chinese going abroad is different from the colonization protected by power in western countries, but a peaceful and civilized immigrant with working people as the main body [4]. The overseas Chinese culture has relative independence, highlighting the gap between Chinese and Western cultures. At the same time, it is also the product of the integration of Chinese and Western cultures, which has not been assimilated into the development process of the world. On the contrary, it can develop and innovate in the torrent of economic exchanges and culture, maintain a free development mode, and become the driving force to promote the further development and self-improvement of overseas Chinese culture, so as to derive a group of overseas Chinese with high knowledge level and strong adaptability and make contributions in the fields of economy, culture, science, and technology [5].

Diversified cultural attributes maintain the original fine traditions of the Chinese nation and quickly absorb the advantages and specialties of other national cultures, so as to enrich and improve their own ability [6].

Overseas Chinese culture is the result of the large-scale overseas migration of Chinese people in modern times, the preservation of broad and profound Chinese culture, and the continuous absorption of the essence of western culture [7]. It has become the product of the exchange and integration of Chinese and Western cultures. Due to the differences in the economy and culture of foreign countries, it is very challenging to be familiar with their economy and culture [8]. Therefore, overseas Chinese must constantly update and change, keep pace with the development of other countries, and, at the same time, organically combine the original unique culture of the Chinese nation with the local culture, so as to make the change trend of the traditional culture of overseas Chinese and the inheritance trend of the traditional culture of overseas Chinese go hand in hand, so as to make them integrate and develop together and maintain the freshness, vitality, and creativity of the overseas Chinese culture [9].

Overseas Chinese culture reflects the humanistic spirit and embodies the noble national spirit and national integrity that inspire contemporary and future generations to work hard and love their country. Chinese traditional culture is impacted by western culture. The new lifestyle and new culture imperceptibly absorb new cultural factors and accept new lifestyles in constant contact, exchange, friction, and conflict so that overseas Chinese can gradually establish the concept of self-confidence and openness and have an all-inclusive attitude. The particularity of historical evolution endows overseas Chinese culture with strong vitality that is good at absorbing the advantages and specialties of other national cultures [10].

## 3. The Development and Reform of Overseas Chinese Culture

The formation and development of overseas Chinese culture is not a process of Westernization. As an ancient civilization with a long history in the world, China has a unique traditional culture [11]. The tradition of “falling leaves and returning to their roots” has not been forgotten and replaced in the development of overseas Chinese culture [12]. Overseas Chinese have formed a culture of constant struggle for self-improvement, retained the traditional virtues of the Chinese nation of hard work and self-reliance, and excavated a strong personality of independent exploration [13]. Overseas Chinese has gradually made remarkable achievements in the economy. The continuous development and reform of overseas Chinese culture has gradually improved the social status of overseas Chinese in foreign countries, made overseas Chinese living in foreign countries more confident and have more voice, driven the healthy and benign development of China's relations with other countries, and connected the development of Chinese enterprises in other countries [14].

Chinese traditional culture itself has the temperament of being implicit, introverted, restrained, and reserved. Confucianism teaches people to learn self-discipline, restrain selfish desires, and abide by etiquette and moral norms. In contrast, most Latin American countries belong to a typical indulgent culture. The contempt for labor and the devaluation of wealth in Catholic ethics may be one of the reasons for this phenomenon. Catholicism opposes people's excessive pursuit of material wealth and condemns those who are greedy for wealth. At the same time, it believes that the purpose of labor is to survive and self-sufficiency and encourages people to be content. The direct reflection of this concept of wealth and labor in today's Latin American society is that compared with work, people pay more attention to leisure and entertainment and have a more casual and relaxed lifestyle and a higher degree of happiness [15].

The integration of immigrants is affected by many factors. This part will use the theory of cultural dimension to analyze the advantages and obstacles of overseas Chinese in the process of integrating into local society from the perspective of cultural values. It should be made clear that Chinese, overseas Chinese, and ethnic Chinese belong to different concepts [16]. Although Chinese immigrants, especially the third generation immigrants, have Chinese descent, they have been partially or completely localized in terms of language, habits, lifestyle, and values, so they have a high degree of social integration. The research object of this paper is mainly the overseas Chinese who were born in China and have lived in China or the second-generation immigrants who were born in the country of residence but have a strong sense of Chinese cultural identity [17].

Both foreign countries' sense of identity with Chinese immigrants and Chinese immigrants' sense of identity with the country of residence are at a relatively low level. Although as an immigrant country, it is the basic national policy of all countries to absorb immigrants, the loose immigration policy is mainly aimed at European immigrants and Asian immigrants, including Chinese, have been discriminated, and excluded to varying degrees for a long time. From the end of the nineteenth century to the first half of the twentieth century, many countries have set off a wave of anti-Chinese many times. After the 1990s, with the rise of China's national strength, the attitude of various countries towards overseas Chinese has also undergone positive changes, and the contribution of overseas Chinese has been more affirmed. However, the stereotype of the status of European and American Chinese as the center of history and culture still exists. Argentine scholars have analyzed the reports on immigration issues published by the two mainstream media with the largest circulation in the country, the national newspaper, and the horn newspaper, from 1999 to 2005. Research shows that when talking about “foreigners in Argentina,” only Latin Americans and Chinese are called “immigrants,” while Europeans and Americans are called “executives,” “professionals,” or “entrepreneurs” [18]. This example shows that the Argentine Society does not treat immigrants from different countries equally. “Immigration” specifically refers to people seeking job opportunities and social promotion, which is derogatory, while groups from European and American countries do not belong to “immigration” because they maintain their original economic and social status [19].

In a society with high uncertainty avoidance, people regard “different things are dangerous,” so they have strong racial prejudice and xenophobia and are more hostile to foreign immigrants. The nationalist tendencies and prejudice against the Chinese in many countries can partially verify this judgment. On the contrary, Chinese immigrants also harbor cultural nationalism, have a strong cultural and emotional identity with China, have a “guest” mentality towards the country of residence, and are used to using “we” and “they” to distinguish their peers and locals. At the same time, they also have a certain prejudice against blacks and Indians in the country of residence. Nowadays, China's food culture, festival customs, traditional Chinese medicine, and Chinese have been widely spread in various countries through the media and bridge of overseas Chinese, attracting the attention and love of more and more people in various countries. Most overseas Chinese have also accepted the local cultural traditions, and the mutual recognition between the two sides has gradually improved [20].

Collectivism culture has two typical manifestations among Chinese and overseas Chinese. First, the family business model is very common. Family ties and acquaintances have played an extremely important role in the process of Chinese immigration. The strong sense of family responsibility not only makes “chain migration” the main migration path of the Chinese but also gives the Chinese economy a strong clan color. When choosing partners or employees, family members and fellow countrymen are given priority. Second, Chinese groups have the strength to seek unity and mutual assistance. Since the late nineteenth century, overseas Chinese in Latin America have established overseas Chinese organizations. Nowadays, all countries have overseas Chinese groups and associations with different numbers, functions, and sizes.

The influence of collectivism also has two sides. On the one hand, both family business and mutual assistance, as well as immigration organizations, help the Chinese to stay together and cope with various difficulties in the process of cultural adaptation. On the other hand, too much emphasis on and reliance on collectivism may also lead to the formation of strong cohesion within the group, resulting in exclusion as “outsiders” by other groups. This relative closeness is manifested in the lack of contact between overseas Chinese groups, their own policies, and even the phenomenon of disunity and exclusion. The external performance is that the Chinese social circle is narrow and single, is limited to the Chinese community, and lacks contact with local people. When studying the new Chinese immigrants in Chiapas, Mexico, domestic scholars found a case in which they can better integrate into the local society after cutting off the connection with the Chinese community. Although this case is not universal, it also proves the importance of the Chinese surpassing and breaking through the original circle of friends, reducing their dependence on each other, and expanding and diversifying their social networks for social integration.

Collectivism has promoted employees to take on a new look, always adhere to strict management, strengthen assessment and accountability, regularly organize and carry out special inspections of discipline style, effectively solve the problems of work procrastination, buck-passing, and out of shape implementation, promote the further reversal of work style, and constantly revise and improve the code of conduct for employees (as shown in Figure 2) according to the actual development of the enterprise.

## 4. Evolution of Overseas Chinese Culture to Chinese Enterprises

In recent years, overseas Chinese have begun to pay extensive attention to political activities, and various types of overseas Chinese associations and organizations have sprung up all over the world. Overseas Chinese have gradually occupied a seat in the political arena of their country and have a certain voice, marking the further improvement of the social status of overseas Chinese. Before the 1970s, the social development trend of overseas Chinese generally showed the trend from falling leaves and returning to roots (overseas Chinese) to taking root (overseas Chinese)—integrating into local society (assimilating into local people), with the characteristics of rapid development and large scale (as shown in Table 2).

### 4.1. The Rise of Chinese Enterprises

With the continuous improvement and consolidation of the status of overseas Chinese in the political and economic fields, overseas Chinese have made remarkable economic achievements, resulting in the emergence of a large number of enterprise groups, which have become an integral part of the local economy. For overseas Chinese who have lived abroad for a long time, they often pay attention to returning to their roots when they are old, living in their hometown, or running enterprises, resulting in a cultural collision and new forms. Since World War II, overseas Chinese culture has undergone a qualitative change, and overseas Chinese culture has been gradually replaced by a new type of Chinese culture. People can see that although most Chinese have joined the local nationality, the code of conduct and values retained from their bones cannot be changed overnight. The traditional overseas Chinese culture has lost its fertile soil of existence by settling abroad from China. Overseas Chinese travel abroad. In addition, the local government does not allow the transplantation and dissemination of culture for the purpose of allegiance to China. Some governments even adopt the policy of forced assimilation to try to eliminate the Chinese culture and completely localize the Chinese culture. This trend makes the overseas Chinese in foreign countries self-improvement. Thus, some seeds have quietly changed in the Chinese mentality, making them change from “falling leaves and returning to roots” to “taking root.”

### 4.2. The Relationship between the Development Opportunity of Chinese Enterprises and the Construction of Enterprise Culture

The “One Belt, One Road” International Cooperation summit opened at the Beijing National Convention Center, which has attracted close attention from overseas Chinese and the overseas Chinese of other countries. One belt, one road has been seen by many overseas Chinese businessmen who have strong capital strength and economic resources. They have seen the new opportunities and new changes in their life under the initiative of “one belt and one road.” Since then, overseas Chinese have become a bridge and link connecting the economy and trade between China and other countries, which is strong support and guarantee for Chinese enterprises to “go global.” One belt, one road initiative will help one belt, one road, and one country along the road. Chinese culture and corporate culture are both organically unified and can be mutually constructed and integrated. According to the four-level structure theory of corporate culture, we can make efforts from the four aspects of spiritual level, institutional level, behavioral level, and material level to promote Chinese culture and corporate culture as mutual means, driving force, bond, and service for each other. Through concept guidance, system integration, behavior orientation and image building continuously promote the smooth realization of the production and operation objectives of the enterprise (as shown in Figure 3), comprehensively shape and improve the corporate culture, and form a cultural system including ideas (as shown in Table 3).

### 4.3. Attach Importance to the Education of Overseas Chinese Culture

The development of the country and economy is inseparable from culture, which is also proved by the continuous development of overseas Chinese culture. Overseas Chinese cultural education not only can provide opportunities for overseas Chinese to learn their own language and inherit the traditional culture of the Chinese nation but also can spread the Chinese language—Chinese on the world stage, making Chinese a bridge and messenger for the exchange and integration of Chinese culture and the language and culture of all nationalities in the world and playing a positive role in promoting the development process of Chinese enterprises. The exchange and integration of languages and cultures between different countries and nationalities, learning from each other's strong points to complement each other's weaknesses, and coexistence for common prosperity are not only problems at the cultural level, but also an important factor affecting the peace and development of today's world. It is the overseas Chinese cultural education that helps overseas Chinese understand the essence of Chinese traditional culture through historical stories and timely, truly, objectively, and accurately convey the actual development status of our country, so as to arouse the sense of national cultural identity and mission of overseas Chinese and then guide overseas Chinese to actively participate in various construction of our country and promote the development of Chinese enterprises.

## 5. The Influence of Chinese Cultural Integration Environment on the Development of Chinese Enterprises

### 5.1. The Influence of Family-Based Thought on the Success of Chinese Enterprises

In the eyes of Chinese people, the family is a small society integrating production, consumption, education, insurance, and life. The family standard thought is the leading spirit of family ethics in Chinese traditional society. The family standard emphasizes the supremacy of family interests, blood relationship, and family harmony. It has a strong exclusiveness and emphasizes the sustainable and long-term development of the family. Throughout the development history of Chinese traditional ethics, the thought of family standards runs through all the time. China has a strong family-based thought, which is formed for two reasons: first, it is determined by the special social structure of ancient China, and second, in China's traditional small-scale peasant society based on self-sufficiency, there is a serious dependence on the family.

Family-based thought is closely related to the success of the Chinese. Most Chinese enterprises in the world are family enterprises. It is an enterprise established and developed on the basis of the family. In China, setting up enterprises and working hard for them are for the benefit of the whole family, for raising families with family property, and for passing on family property to future generations. Chinese people's property is more used for saving; the West is more willing to entrust enterprises to outsiders; and timely consumption is the motivation of enterprise development. In addition, in order to increase family assets and pursue maximum profits, the Chinese invest their funds in industries with high profits and withdraw from industries with low profits. In the West, the development of enterprises is for the development and growth of enterprises themselves.

Under the influence of the concept of family standard, although Chinese family enterprises occupy a place in the world and there are many world-class tycoons among Chinese, there are still some obstacles to their development. For example, it takes its own family members as managers, which makes it difficult for Chinese family enterprises to embark on institutionalized management. It implements the property distribution system of the combination of unification and division, not the eldest son inheritance system, which makes the equity responsibility of the enterprise unclear. For these obstacles, Chinese family enterprises need to optimize the management system, absorb the management elite into the management, and constantly learn and adapt to the marketing model of cross-cultural management (as shown in Figure 4).

### 5.2. The Influence of Chinese Traditional Philosophy of Emphasizing Agriculture and Restraining Business on the Success of Chinese Enterprises

The conceptual organization is conducive to managers' correct analysis and decision-making in the management process by virtue of the organization type structure and the characteristics of high dependence on knowledge and ability (as shown in Figure 5).

In addition, China's traditional philosophy of emphasizing agriculture and restraining business also has a great impact on the success of Chinese enterprises. In ancient times, businessmen were rarely encouraged by the government, and their capital was almost evenly distributed. Therefore, many household products were consumed by themselves. The policy of emphasizing agriculture and restraining commerce was formed in the pre-Qin period. Mencius and Legalists of Confucianism put forward such an idea. It developed in the Qin and Han dynasties. Shang Yang's reform opened the precedent for its development. The policy of emphasizing agriculture and restraining business is the reflection of the natural economy and the inevitable product of the low level of social productivity. The essence of the policy of emphasizing agriculture and restraining commerce is to safeguard the feudal economic foundation, safeguard the interests of the landlord class, and consolidate their own rule. Although this policy has promoted the prosperity and development of the agricultural economy to a certain extent, mobilized the enthusiasm of farmers, and is conducive to the prosperity and development of the economy, it has also brought many negative effects. For example, this policy has restrained the development of the commercial economy, made enterprises only stay within the family, and laid a foundation for Chinese family enterprises to expand their relations from within their own family, which cannot surpass the family and establish a modern enterprise management model. In addition, this policy also makes the development of Chinese enterprises lack the spirit of constitutionalism. Even if it makes Chinese enterprises based on development in the world, it also brings many problems, such as the management system and model cannot keep pace with the times.

In short, the family system with the profound historical origin and cultural precipitation is the foundation of supporting Chinese society and has a profound impact on China's development for thousands of years. The ethical concept of family standard based on a self-sufficient family society, the traditional philosophical thought of emphasizing agriculture and restraining business, and the traditional thought of “being an official and making money” all play a positive role in the development of Chinese enterprises.

## 6. Conclusion

First of all, values are the deepest expression of culture, and cultural differences have many forms of expression. In many cases, people see its external side. Secondly, different races, religions, genders, generations, and classes have different cultural characteristics, which only reflect part of the national (regional) cultural dimension, not all. Thirdly, the correlation between cultural dimensions is different in different countries (regions), which leads to obvious differences in the specific practical activities of countries (regions) close to one dimension due to the different influences of other dimensions. The influence of cultural values on the social integration environment of overseas Chinese is the focus of this paper. As for other influencing factors, such as the immigration environment and immigration policy of the country where the overseas Chinese live, the cultural literacy and social background of the overseas Chinese, and how the overseas Chinese overcome the obstacles and realize cross-cultural adaptation, it needs to be further studied in the future. On the whole, the cultural differences between China and Latin America have caused great obstacles to the cultural adaptation and social integration of the Chinese. This is the same dilemma faced by immigrant groups around the world. However, in some cases, cultural differences are not necessarily a bad thing. For example, the degree of the economic integration of Chinese in Latin America is relatively high. In any case, the integration of immigrants is a long process, and cultural values are an important influencing factor.

The degree of social integration of immigrants is affected by many factors. Western scholars pay more attention to explaining the discrimination, exclusion, or restriction of immigrants in the host country from the perspective of objective conditions such as system, human capital, and social capital, which is mainly based on people's cognition of the poor integration of immigrants in the inflow place. The ultimate purpose of the study is to promote countries to formulate policies conducive to the integration of migrants, so as to improve and improve the integration of migrants. However, it is obvious that the social integration of immigrants is also affected by the differences between their own culture and the culture of the country where they live, and this influence runs through the whole process and all stages of social integration, with far-reaching and lasting characteristics. When studying the social integration of Chinese and overseas Chinese, domestic scholars generally believe that the cultural differences between China and foreign countries and the resulting embarrassment of cross-cultural communication are the biggest obstacle for Chinese immigrants to integrate into local society. For example, when studying the social integration of Chinese in Australia, some scholars believe that “cultural differences are doomed that Chinese cannot be fully assimilated by Australian society.” When studying the social integration of Chinese in South Africa, some scholars believe that “cultural differences and utilitarian “passers-by” adaptation strategies have affected the long-term development of new Chinese immigrants in South Africa to a certain extent.” It can be seen that culture is a very important factor in the social integration of overseas Chinese.

If the overseas Chinese culture has experienced the whole process of collision, identification, assimilation, selection, and innovation, then the traditional overseas Chinese culture has experienced the process of collision, identification, and assimilation. Wang Kangmei believes that if Chinese culture has experienced the whole process of collision, identification, assimilation, selection, and innovation, then Chinese enterprises have also experienced corresponding development, which is consistent with the point of view in the article. There is an old Chinese saying that “the kindness of a drop of water should be rewarded by a spring.” In the process of continuous self-charging and self-strengthening, overseas Chinese have not forgotten the root but continuously strengthened and deepened the Chinese civilization and Chinese spirit on the global stage. Many years ago, many Italians had to sell their business to the Chinese because of business difficulties. Now, the Chinese not only use their wisdom and diligence to carry forward their business step by step but also give back to the country with a grateful heart. This is a good phenomenon. It shows that the strength of the motherland has affected overseas, the national self-confidence has been greatly strengthened, and the cultural self-esteem has been improved. The return of Chinese enterprises illustrates that the essence of Chinese culture has gone deep into the hearts of every Chinese people. The development of overseas Chinese culture to Chinese enterprises enables other countries in the world to better understand, know, yearn for, and feel China.

## Figures and Tables

**Figure 1:** Four-level structure model of overseas Chinese culture.

**Figure 2:** Employee code of conduct.

**Figure 3:** Mutual construction and integration of Chinese culture and corporate culture.

**Figure 4:** Mutual construction and integration of Chinese culture and corporate culture.

**Figure 5:** Cultural integration model.

**Table 1:** Definition of corporate culture.

Scholars	Definition of corporate culture
Hofstede	The mental process of an organization
Deere and Kennedy	The main values that the organization believes in
Peters and Waterman	The values that all employees abide by together, that is, the rules of conduct that are acceptable to all
Dennison	Value, belief, and behavior pattern, the core identity of an organization

**Table 2:** Seven Chinese rich in Forbes 2013 Thailand's top 10 rich list.

Rank	Name/family	Net assets	The main group company
1	Dhanin Chearavanont and his family (Dhanin Chearavanont and family)	126	Bobi group
2	Zheng Youying family (Chirathivat family)	123	Central group
Central Group3	Su Xuming (Charoen Sirivadhanabhakdi)	106	TCC group
4	Xu Shubiao family (Yoovidhya family)	78	Red Bull Thailand Company
5	Li Zhizheng	39	Dacheng Bank
8	Xu Hanguang and his family (Vichai Maleenont and family; Krit Ratanarak)	20	BEC World Group
10	Thaksin Sinawatra and his family (Thaksin Shinawatra and family)	17	Qinnayue Computer Telecom Group

**Table 3:** Corporate philosophy and culture system.

Enterprise vision	First-class production enterprises in China
Enterprise philosophy	Be sincere in believe and be far away
Enterprise strategy	Expand the brand and strengthen the enterprise
Entrepreneurship spirit	Pragmatic innovation passion surpasses
Enterprise style	Strict, fine, and solid
Talent concept	Cultivate the position of cultivating talents, compete, and choose talents
Learning idea	Learn ability + innovation ability = competitiveness
Concept of quality and safety environment	Strive for perfection, pursue perfection, provide high-quality service, create satisfaction, comply with the law, be safe, optimize the environment, strive for continuous improvement

## Data Availability

The labeled data set used to support the findings of this study is available from the author upon request.
